# Inhibited corneal neovascularization in rabbits following corneal alkali burn by double-target interference for VEGF and HIF-1α

**DOI:** 10.1042/BSR20180552

**Published:** 2019-01-30

**Authors:** Ying-Cong Fu, Zhi-Ming Xin

**Affiliations:** Department of Burns and Plastic Surgery, Shengli Oilfield Central Hospital, Dongying 257034, P.R. China

**Keywords:** Alkali burn, Cornea neovascularization, Gene silencing, HIF-1α, Rabbit model, Synergistic effect, VEGF

## Abstract

Expression of hypoxia-inducible factor (HIF) 1α has been observed in corneal neovascularization (CNV). Vascular endothelial growth factor (VEGF), one of the most well-known angiogenic factors in CNV, is under the regulation of HIF-1. The present study aims to investigate the synergistic effects of VEGF and HIF-1α gene silencing on alkali burn-induced CNV in rabbits. The models of rabbits in corneal alkali burn were established. SiRNA recombinant adenovirus was used to explore the synergistic effects of VEGF and HIF-1α gene silencing on alkali burn-induced CNV. CNV area and ultrastructure of cornea were observed. The expression of VEGF and HIF-1α was detected. CNV was observed in rabbits following alkali burn. In addition, overexpressed VEGF and HIF-1α was also observed in rabbits following alkali burn. Then, silencing HIF-1α or silencing VEGF decreased area of CNV, inhibited neovascularization and improved pathological changes, while double-target interference for VEGF and HIF-1α decreased area of CNV inhibited neovascularization, and improved pathological changes to a greater extent. Our study provides evidences emphasizing the distinct notion that VEGF and HIF-1α play the contributory role in alkali burn-induced CNV as a result of double-target interference for VEGF and HIF-1α inhibiting CNV in rabbits following corneal alkali burn.

## Introduction

Normal cornea is transparent and free of blood vessels, and corneal avascularity is critical for optical clarity and maintenance of vision [1]. Corneal neovascularization (CNV) is considered as a sight-threatening condition, which is marked by corneal ingrowth of new blood vessels, and typically correlated with toxic, infectious, inflammatory, traumatic, immunological, or degenerative disorders of the cornea and ocular surface [2,3]. Therefore, ophthalmic diseases represented by CNV are considered as a major public health hazard [1]. Under the conditions of corneal infections, misuse of contact lens, chemical burn, and inflammation, the vascularization of normal cornea often occurs owing to the disequilibrium between angiogenic and antiangiogenic stimuli, which leads to a surplus of proangiogenic factors like vascular endothelial growth factor (VEGF) [4,5]. Alkali burn is regarded as one of the most serious contributors of CNV and may cause severe injury to the cornea and vision [6]. Some treatments, such as laser photocoagulation, medication, and surgery, are applied for the treatment of CNV diseases, but recently, no clear consensus has been reached on the most efficacious treatment option for CNV, which indicates that novel treatments for CNV diseases are in urgent need [7,8].

VEGF, a member of the platelet-derived growth factor supergene family, serves as a crucial participator in stimulating the multiplication of endothelial cells and formation of new blood vessels [9]. As one of the primary proangiogenic factors of both physiological and pathological angiogenesis, the up-regulation of VEGF is maintained during diverse forms of pathological angiogenesis [10]. Moreover, VEGF silencing has shown potential for CNV treatment via directly inhibiting the angiogenesis at a molecular level [8]. Hypoxia-inducible factor (HIF)-1α is a subunit of the transcription factor HIF-1, which is a heterodimer, composed of an α and a β subunit [11]. Under hypoxic conditions, HIF-1α plays a critical role in vascular remodeling, the products of which are involved in angiogenesis, erythropoiesis, energy metabolism, and cell survival [12]. Very few studies have covered the synergistic effect of VEGF and HIF-1α gene silencing on CNV. It has been demonstrated that increased expression of HIF-1α and VEGF-B can promote vasculogenesis [13]. Yang et al. [14] reported that VEGF is the most well-characterized angiogenic factor in CNV regulated by HIF-1. In order to investigate whether these double gene silencing will function in alkali burn-induced CNV, rabbits were used in the present study.

## Materials and methods

### Ethics statement

All animal experiments were approved by the animal research ethics committee of Shengli Oilfield Central Hospital.

### Construction of recombinant adenovirus

Purchased from American Type Culture Collection (ATCC, VA, U.S.A.), pAd adenovirus vectors were respectively synthesized into two complementary pairs of specific siRNA targetting rabbit *HIF-1α* mRNA (NM001082782) and rabbit *VEGF* mRNA (serial number: AB020216) by Ribo Biotechnology Co., Ltd. (Guangzhou, China). The synthetic sequences were shown in Table 1. After the formation of dsRNA by annealing, the synthetic sequences were cloned to pSUPER inference vectors linked up with pAdTrack by enzyme digestion, and transferred in the competent bacteria BJS183 containing pAdEasy-l for recombination. A small amount of plasmid DNA of transformed cloned bacteria was extracted and plasmid DNA of suspicious recombinant adenovirus was identified by restriction enzyme digestion. The successfully identified pAd-HIF-1α, pAd-VEGF, pAd-HIF-1α-VEGF, pAd-NC (negative control) were used for the packaging and amplification of recombinant adenovirus vectors.

**Table 1:** siRNA sequences for construction of recombinant adenovirus

siRNA	Sequence
HIF-1α siRNA	Forward: 5′-UACGUUGUGAGUGGUAUUAUUDTDT-3′
	Reverse: 5′-DTDTAUGCAACACUCACCAUAAUAA-3′
VEGF siRNA	Forward: 5′-UCGAGACCUUGGUGGACAUDTDT-3′
	Reverse: 5′-AUGUCCACCAAGGUCUCGADTDT-3′
NC siRNA	Forward: 5′-UUCUCCGAACGUGUCACGUDTDT-3′
	Reverse: 5′-ACGUGACACGUUCGGAGAADTDT-3′

### Establishment of model of rabbit with corneal alkali burn

A total of 54 New Zealand purebred white rabbits (male and female) aged 2–3 months and weighed between 1.5 and 2.0 kg were purchased from Shandong Academy of Agricultural Sciences (Jinan, China). The cornea of each rabbit was normally observed under the slit lamp microscope and those with any ophthalmic diseases were excluded. The rabbit model of corneal alkali burn was established [15]. Before operation, the rabbits were anesthetized by injecting with 30 g/l pentobarbital sodium (30 mg/kg) via ear vein. Tetracaine eye drops (5 g/l) were dropped into the right eye twice, and a cotton swab was used to remove conjunctival sac fluid. Single circular filter paper with a diameter of 8 mm was immersed in 1 mol/l sodium hydroxide solution. One minute after saturation, cotton swab was used to wipe off excess liquid. When the filter paper was placed on the central cornea of each rabbit’s right eye for 1 min, it was removed. Normal saline was used to fully wash the rabbits’ conjunctival sac for 1 min. For the left eye of all rabbits, normal saline was the substitute for the sodium hydroxide solution, as a self-control group. The recombinant plasmid, after subconjunctival injection, was divided randomly into six groups with nine rabbits in each group, including normal control group, blank group, NC siRNA group, HIF-1α siRNA group, VEGF siRNA group and HIF-1α-VEGF siRNA group. In the normal control group, 0.3 ml normal saline was injected into the conjunctivas of normal rabbits. In the blank group, 0.3 ml normal saline was injected into the alkali-burned rabbits’ conjunctivas. In the NC siRNA group, 0.3 ml NC pAd-NC adenovirus (5 × 10^8^ pfu/ml) was injected into the alkali-burned rabbits’ conjunctivas. In the HIF-1α siRNA group, 0.3 ml pAd- HIF-1α adenovirus (5 × 10^8^ pfu/ml) was injected into the alkali-burned rabbits’ conjunctivas. In the VEGF siRNA group, 0.3 ml pAd-VEGF recombinant adenovirus (5 × 10^8^ pfu/ml) was injected into the alkali-burned rabbits’ conjunctivas. In the HIF-1α-VEGF siRNA group, 0.3 ml pAd-HIF-1α-VEGF adenovirus was injected into the alkali-burned rabbits’ conjunctivas. The growth of CNV of rabbits were observed on days 1, 7, and 14 by TopconSL8z slit lamp microscope (Japanese Topcon Inc., Tokyo, Japan) and the growth area of the CNV was calculated and recorded.

### Corneal observation by confocal microscopy

After the alkali-burned rabbits were anesthetized, the biepharostat was used to open the eyelids of rabbits and the vidisic ophthalmic gel was dropped into the eyes of rabbits. After the height of laboratory console and the position of camera were adjusted, the surface of microscope was added with a drop of vidisic ophthalmic gel and then covered by disposable sterile contact cap of cornea. The eyes of rabbits were fixed on the microscope to observe the number and morphological change of corneal cells.

### Hematoxylin–Eosin staining

The rabbits were killed by random air embolism method on days 1, 7, and 14 after burning by alkali, and then the corneal tissues of 1-mm wide sclera were removed. The removed corneal tissues were quickly soaked in 4% paraformaldehyde solution and fixed (at least 24 h) in darkness, dehydrated with gradient ethanol, and then paraffin-embedded. The tissues were cut into serial coronal section with a thickness of 5 μm in a direction which was approximately in parallel with the optical axis. Placed on slides, the sections were baked in an oven at 80°C for 5 min and dewaxed by xylene twice (10 min/time). The sections were rinsed and differentiated in ethanol with concentrations of 100, 95, 75, and 50%, respectively, washed by water, stained in Hematoxylin for 10 min, rinsed for 15 min in water, stained in Eosin for 30 s and cleaned by double-distilled water to wash the extra Eosin away. After dehydration by ethanol and clearing by xylene, the sections were sealed with neutral balsam, and then observed and photographed under a microscope (Olympus BX61; Olympus; Suzhou Rocky Optical Co. Ltd., China).

### Immunohistochemistry

The paraffin sections were placed in a constant temperature oven at 60°C for drying, and after 24–48 h, sections were dewaxed by xylene two times (10 min for each). The sections were dehydrated by gradient ethanol, rinsed using distilled water for 5 min and PBS for approximately 5 min, and then added with 3% hydrogen peroxide solution. Incubated at room temperature for 10 min, the sections were rinsed with PBS three times (3 min for each). Then the sections were added with citric acid buffer solution (pH 6.0), placed in a microwave oven for 20 min, and rinsed by PBS for three times (3 min for each). Normal goat serum was added and the sections were incubated at room temperature for 5 min. After the serum was removed, sections were added with the diluted mouse anti-rabbit HIF-lα monoclonal antibody (1:20, ab2771, Abcam Company, Cambridge, MA, U.K.) and the diluted mouse anti-rabbit VEGF monoclonal antibody (1:200, ab1316, Abcam Company, Cambridge, MA, U.K.), incubated at room temperature overnight and rinsed with PBS three times; 30 μl biotin-labeled goat anti-mouse secondary antibody (1:500, ab97023, Abcam Company, Cambridge, MA, U.K.) was added. The sections were incubated at room temperature for 15 min and rinsed with PBS three times (3 min for each time). Next, sections were added with streptavidin (peroxidase)-labeled streptomycin ovalbumin working fluid, incubated at room temperature for 15 min, and rinsed with PBS for approximately three times (3 min for each time). Sections were developed by adding with the freshly prepared DAB solution (ENS000, Simpson Biotechnology Co. Ltd., Shanghai, China), observed under microscope for 3–5 min, and then rinsed with tap water. Re-stained by Hematoxylin, the sections were washed with tap water again. Ethanol with concentrations of 50, 75, 95, 100% and xylene, respectively, were used for section dehydration (each for 5 min). Sealed with neutral balsam, the sections were observed and photographed under the light microscope. PBS replaced the primary antibody as the NC group, and the other experimental steps were the same as above. The positive expression of HIF-1α was epitomized by yellowish-brown particles in the nucleus. The positive expression of VEGF was epitomized by yellowish-brown or brown granules in cytoplasm. Each section was observed from five randomly selected visual fields under the high magnification microscope (×400), and the images were collected by the high definition color pathological image analysis system (HMI AS-2000, Wuhan Champion Image Technology Co., Ltd., Wuhan, China), and analyzed by Image-Pro Plus 6.0 image analysis software (Media Cybernetics Co., Ltd., U.S.A.).

### Reverse transcription quantitative PCR

Rabbits were killed by air embolism method on the 1st, 7th, and 14th days after alkali burn, and the corneas were excised from limbal cornea at 0.15 mm position under sterile conditions. The total RNA was extracted by the RNA Extraction Kit (BioTeke Corporation, Beijing, China) using TRIzol method (Invitrogen, CA, U.S.A.) and then kept at −80°C. The total RNA was reversely transcribed to cDNA by Prime Script^®^ RT reagent Kit (Perfect Real Time) (Takara, Tokyo, Japan), and the reverse transcription reaction conditions were as follows: at 37°C for 15 min and at 85°C for 5 s. Then the transcribed cDNA was stored at −20°C. The reverse transcription quantitative PCR (RT-qPCR) experiment was performed by the application of ABI 7500 qPCR (ABI, U.S.A.). The primer sequences were shown in Table 2, and the amplification reaction conditions were as follows: 1 cycle for 10 s at 95°C, 40 cycles for 5 s at 95°C and for 30 s at 60–61°C. The reaction systems were: 12.5 μl Premix ExTaq or SYBR Green Mix, 1 μl Forward Primer, 1 μl Reverse Primer, 1–4 μl DNA template, and 25 μl ddH_2_O. PCR products were identified by 1% agarose gel electrophoresis. The data were analyzed by 2^−ΔΔ*C*^_t_ method, and the formula was as follows: ΔΔ*C*_t_ = [*C*_t_ (target gene) − *C*_t_ (reference gene)] _experimental group_ − [*C*_t_ (target gene) − *C*_t_ (reference gene)] _control group_. The experiment was repeated three times.

**Table 2:** Primer sequences for RT-qPCR

Gene	Sequence
*HIF-1α*	Forward: 5′-GATGGTGCTAACAGATGACGGC-3′
	Reverse: 5′-AGCGGCCCAAAAGTTCTTCC-3′
*VEGF*	Forward: 5′-CTTGCTGCTCTACCTCCACC-3′
	Reverse: 5′-CTTTGGTCTGCATTCACATTTG-3′
*β-actin*	Forward: 5′-CTACAATGAGCTGCGTGTGG-3′
	Reverse: 5′-TAGCTCTTCTCCAGGGAGGA-3′

### Western blot analysis

The corneas of rabbits in each group were collected on the 1st, 7th, and 14th days, respectively, and then added with protein lysate solution (Beyotime Biotechnology Co. Ltd., Shanghai, China) to extract total protein. The extracted proteins were used for SDS/PAGE, and the sandwich-like combination of filter paper–glue film–filter paper was immersed in the buffer solution to transfer the proteins into PVDF membrane (Jiangsu Jie Lv Mo Technology Co., Ltd). The PVDF membranes were blocked in 5% skim milk for 1.5 h with mouse anti-rabbit VEGF primary antibody (1:500, Abcam Inc., Cambridge, MA, U.S.A.), mouse anti-rabbit HIF-1α primary antibody (1:4000, Abcam Inc., Cambridge, MA, U.S.A.), and β-actin primary antibody (1:500, Abcam Inc., Cambridge, MA, U.S.A.) were added respectively. Incubated at 37°C for 2 h, the PVDF membranes were washed with TBS with Tween-20 (TBST) three times (5 min for each). The secondary antibody (1:10000, Abcam Inc., Cambridge, MA, U.S.A.) labeled with horseradish peroxidase (HRP) was added to the PVDF membranes at room temperature. Incubated at room temperature for 2 h, the membranes were washed three times (5 min for each) and developed by chemiluminescence reagent. The β-actin was taken as an internal reference and the Bio-Rad Gel Dol EZ imager (Gel Doc EZ Imager, Bio-Rad, California, U.S.A.) was used for color development. The concentration of β-catenin protein in cytoplasm and nucleus was detected by BCA protein assay kit (P0009, Shanghai Beyotime Biotechnology Co., Ltd., Shanghai, China). Other Western blotting bands were analyzed by gel electrophoresis imaging system (MSD-2000, Beijing MAISIQI High-Tech Co., Ltd., Beijing, China) to conduct analysis of relative optical density, and the β-actin protein was used for calibration amongst groups.

### Statistical analysis

Statistical analysis was performed using SPSS 21.0 statistical software (IBM Corp. Armonk, NY, U.S.A.). Enumeration data were presented in rate and percentage. Chi-square test was used to make comparisons amongst groups. Measurement data were presented as mean ± standard variance. The one-factor ANOVA was used to compare the differences amongst groups (detected by Homogeneity of variance before analysis) and a *P*-value <0.05 indicated statistical significance.

## Results

### Double-target interference for VEGF and HIF-1α significantly inhibits neovascularization in the corneas following alkali burn

Initially, the slit lamp microscope was used to observe the corneas to explore the effect of VEGF and HIF-1α on neovascularization. The experimental results on the 14th day were the most clear. In the normal control group, the corneas were smooth and transparent with no CNV found. In the HIF-1α-VEGF siRNA group, the rabbits showed a large area of transparent corneas, regional slight opacity and a small area of CNV (*P*<0.05). There was no marked difference of the corneas of rabbits between the HIF-1α siRNA and VEGF siRNA groups, in which a large area of semitransparency and local corneal edema existed and a relatively large amount of new vessels extended into the corneal graft. Compared with other groups, the difference between the HIF-1α siRNA and groups was evidently significant (*P*<0.05). No marked difference was found between the blank and NC siRNA groups, in which the corneal edemas of alkali-burned corneas were obvious and lots of new vessels emerged and the experimental results were significantly worse than those of other groups (*P*<0.05). The results of comparisons amongst six groups showed that the area containing CNV in the normal control group was the lowest at every time point and in the HIF-1α-VEGF siRNA group was the second lowest, indicating significant difference (*P*<0.05). There was no clear difference in the areas of CNV between the VEGF siRNA group and HIF-1α siRNA group, but the areas of CNV in the blank and NC siRNA groups were significantly higher than those in the VEGF siRNA and HIF-1α siRNA groups (*P*<0.05). No marked difference was found when comparing the blank group and the NC siRNA group (Figure 1 and Table 3). The aforementioned results reveal that when HIF-1α and VEGF are silenced at the same time, neovascularization in the corneas of rabbits after alkali burn can be suppressed to a greater extent.

**Figure 1:** Under the slit lamp microscope, double-target interference for VEGF and HIF-1α significantly inhibits neovascularization in corneas (**A**) The experimental results on the 14th day after alkali burn under slit lamp microscope; (**B**) the area of CNV of rabbits after alkali burn in each group. *, *P*<0.05 compared with the normal group; ^#^, *P*<0.05 compared with the HIF-1α-VEGF siRNA group; ^&^, *P*<0.05 compared with the HIF-1α siRNA group.

**Table 3:** The lengths of CNV of rabbits after alkali burn (mean ±S.D.)

	Eyes (*n*)	Normal control	HIF-1α-VEGF siRNA	HIF-1α siRNA	VEGF siRNA	NC siRNA	Blank
Length (mm)	9	0.00 ± 0.00	0.21 ± 0.05	2.3 ± 0.80*	2.4 ± 0.70*	3.2 ± 0.40*	3.1 ± 0.50

* *P* < 0.05 compared with the normal group.

### Double-target interference for VEGF and HIF-1α promotes the healing of corneal epithelial cells and inhibits inflammatory cell infiltration

The confocal microscopy was applied to observe the ultrastructure of corneas of rabbits after alkali burn. The results showed that on the 1st day after alkali burn, the corneas of rabbits in each group occurred corneal epithelial cells swelling, the nucleus presented blurry, loosely arranged, disordered and incomplete, and the corneal epithelial cells in partial regions occurred single-layer deletion or complete deletion with lumps occurred and the high reflective light regions of cell structure were indistinguishable. On the 7th day after alkali burn, the rabbits in the blank group showed CNV in corneal limbus and the vessels were thin and tortuous. The rabbits in the HIF-1α-VEGF siRNA, HIF-1α siRNA, and VEGF siRNA groups showed small amount of CNV and thin vessels. On the 14th day, the corneal epithelium of rabbits in the blank group basically healed, the corneal epithelial cells presented pentagonal or hexagonal forms again, while partial deleted corneas stile occurred a small amount of inflammatory cell infiltration. In the HIF-1α-VEGF siRNA, HIF-1α siRNA, and VEGF siRNA groups, the deleted corneal epithelial cells of rabbits showed good healing without any inflammatory cell infiltration (Figure 2). From these findings, it can be inferred that silenced HIF-1α and VEGF could improve the corneal epithelial cells healing and reduce inflammatory cell infiltration.

**Figure 2:** Under the confocal microscopy (×800), double-target interference for VEGF and HIF-1α promotes the healing of corneal epithelial cells and inhibits inflammatory cell infiltration in rabbits after alkali burn The results of the corneas on the 1st, 7th, and 14th days after alkali burn observed under the confocal microscopy with the field of vision of 400 μm × 400 μm and the resolving power of 1 μm.

### Double-target interference for VEGF and HIF-1α significantly improves pathological changes in alkali-burned corneal tissues

Hematoxylin–Eosin (HE) staining was conducted to observe pathological changes in alkali-burned corneal tissues, and the results of corneal pathological sections were the clearest on the 14th day. In the normal control group, the epithelium, Bowman’s layer, substantia propria, Descemet’s membrane, and endothelium of rabbit corneas were well organized with almost no inflammatory cell infiltration. A small amount of inflammatory cell infiltrations were seen in the HIF-1α-VEGF siRNA group, with few and scattered narrow blood vessels, and the severity of results was between those of the normal control group and the single-gene interference groups (the HIF-1α siRNA group and the VEGF siRNA group). In the VEGF siRNA and HIF-1α siRNA groups, there were a large number of infiltrated inflammatory cells in the substantia propria, mostly polymorphonuclear leukocytes, and much new vessels in the Bowman’s layer. In the blank and NC siRNA groups, a lot of inflammatory cells infiltrated in the cornea stroma, polymorphonuclear leukocytes, and lymphocytes were relatively abundant, and the inflammatory reaction was strong. Arranged closely, the lumen of mature CNV was enlarged and thickened in the cornea stroma (Figure 3). These results reveal that the aforementioned results reveal that when HIF-1α and VEGF are silenced at the same time, pathological changes in alkali-burned corneal tissues can be improved to a greater extent.

**Figure 3:** HE staining reveals that double-target interference for VEGF and HIF-1α significantly improves pathological changes of corneal tissues on the 14th day after alkali burn The neovascularization containing erythrocyte in the corneal stroma was expressed by black arrowhead, and the corneal stroma presented as edema and mononuclear inflammatory reaction.

### Double-target interference for VEGF and HIF-1α decreases the positive expression of VEGF and HIF-1α in alkali-burned corneal tissues

Next, to explore the effect of VEGF and HIF-1α on alkali-burned corneal tissue, immunohistochemistry was conducted to examine the positive expression of HIF-lα and VEGF. The positive expression of VEGF was evidenced by brown or brown-yellow granules in cytoplasm. The positive expression of HIF-lα was evidenced by brown-yellow and granule-like in the nucleus. According to the final staining degree, the results were divided into: + (weak positive), ++ (positive), +++ (strong positive). The results of immunohistochemistry showed that almost no positive expression of VEGF and HIF-1α expression was seen in the normal control group. Compared with the normal group, the blank group showed higher positive expression VEGF and HIF1α (*P*<0.05). No significant difference in the positive expression VEGF and HIF-1α was found between the blank and NC groups. Compared with the blank group, the HIF-1α-VEGF siRNA and VEGF siRNA groups showed decreased positive expression of VEGF, and the HIF-1α-VEGF siRNA and HIF-1α siRNA groups showed decreased positive expression HIF-lα, indicating a significant difference (*P*<0.05) (Figure 4). All these results revealed that silenced HIF-1α and VEGF reduced the positive expression of VEGF and HIF-1α in alkali-burned corneal tissues.

**Figure 4:** Double-target interference for VEGF and HIF-1α decreases the positive expression of VEGF and HIF-1α in alkali-burned corneal tissue (**A**) The positive staining in each group; (**B**) the positive expression of VEGF and HIF-1α in corneas were examined by immunohistochemistry. *P<0.05 compared with the normal group; ^#^*P*<0.05 compared with the HIF-1α-VEGF siRNA group; ^&^*P*<0.05 compared with the HIF-1α siRNA group.

### Double-target interference for VEGF and HIF-1α reduces the mRNA and protein levels of VEGF and HIF-1α in alkali-burned corneal tissue

Finally, to further investigate the mechanism of VEGF and HIF-1α in neovascularization, RT-qPCR and Western blot analysis were conducted to detect the mRNA and protein levels of VEGF and HIF-1α. The results of RT-qPCR revealed that the mRNA expressions of VEGF and HIF-1α were the lowest in the normal control group and the second lowest in the HIF-1α-VEGF siRNA group. No obvious difference was found between the VEGF siRNA and HIF-1α siRNA groups, in which the expression of *VEGF* mRNA and *HIF-1α* mRNA were clearly lower than those in the blank and NC siRNA groups (*P*<0.05). No obvious difference was found between the blank group and the NC siRNA group (Figure 5).

**Figure 5:** RT-qPCR reveals that double-target interference for VEGF and HIF-1α reduces mRNA expression of VEGF and HIF-1α in corneal tissues after alkali burn (**A**) mRNA expression of VEGF; (**B**) mRNA expression of HIF-1α. *P<0.05 compared with the normal group; ^#^*P*<0.05 compared with the HIF-1α-VEGF siRNA group; ^&^*P*<0.05 compared with the HIF-1α siRNA group.

The results of Western blot analysis showed that protein level of VEGF and HIF-1α were the lowest in the normal control group and the second lowest in the HIF-1α-VEGF siRNA group. No obvious difference was found between the VEGF siRNA group and the HIF-1α siRNA group, and the protein level of VEGF and HIF-1α in the VEGF siRNA and HIF-1α siRNA groups were both significantly lower than those in the blank and NC siRNA groups (*P*<0.05). No obvious difference was detected between the blank group and the NC siRNA group (Figure 6).

**Figure 6:** Western blot analysis demonstrates that double-target interference for VEGF and HIF-1α reduces the protein level of VEGF and HIF-1α in corneal tissues after alkali burn (**A**) Protein bands and protein level of VEGF in corneal tissues after alkali burn; (**B**) protein bands and protein level of HIF-1α in corneal tissues after alkali burn. *P<0.05 compared with the normal group; ^#^*P*<0.05 compared with the HIF-1α-VEGF siRNA group; ^&^*P*<0.05 compared with the HIF-1α siRNA group.

The above results demonstrate that silenced VEGF and HIF-1α reduced the mRNA and protein levels of VEGF and HIF-1α in alkali-burned corneal tissues.

## Discussion

CNV is the most common cause of blindness, which is closely correlated to corneal inflammation, corneal trauma, and corneal allograft rejection [10]. The mechanism of CNV is not fully understood, and even if there are many therapeutic methods, the effects are still not ideal [16]. Therefore, the aim of this study was to investigate synergistic effects of VEGF and HIF-1α gene silencing on alkali burn-induced CNV in rabbits. And the collective results showed strong evidence that VEGF and HIF-1α gene silencing acted synergistically to inhibit CNV.

Initially, it was observed that most corneas in the HIF-1α-VEGF siRNA group were transparent with local mild opacitas, and the area of CNV was very small. However, the area of neovascularization was larger, and the cornea was translucent with local edema in the HIF-1α siRNA group and VEGF siRNA group. According to a previous study, RNAi is an effective gene silencing technique and VEGF siRNA is evidenced to reduce ocular neovascularization [17]. VEGF can contribute to the proliferation and migration of vascular endothelial cells and the increase in the vascular leakage [18–20]. Correspondingly, Zuo et al. reported that in mice with neovascularization induced by alkali burn, siRNA targetting VEGF was beneficial to reduce the expression of VEGF, vascular area, and the number of new vessels [21]. HIF-1α also functions as a regulator in many metabolic pathways, such as vascular tone, cell proliferation, and apoptosis [22]. Overexpression of HIF-1α is related to the increased patient mortality in human cancers, particularly in cancers of the bladder, brain, breast, cervix, endometrium, oropharynx, lung, skin, and stomach, which manifests the inhibition of HIF-1α is crucial in the treatment of many diseases including corneal diseases [23]. Berger et al. [24] supported that HIF-1α inhibition could decrease diseases and corneal destruction.

Besides, HE staining showed that in the HIF-1α siRNA group and VEGF siRNA group, the inflammatory cell infiltration in the corneal stroma was more severe than that in the HIF-1α-VEGF siRNA group. It is reported in a previous study that HIF-1α is an important regulator of immune and inflammatory responses which include nasal symptoms, inflammatory cell infiltration, and eosinophil recruitment [25]. Likewise, VEGF-A was reported to be effective in decreasing both angiogenesis and inflammation [26]. Chang et al. [5] also believe that VEGF increases vascular leakage and promotes monocyte chemotaxis as well as B-cell production in mice, which indicates the significance of VEGF in inflammation.

Immunohistochemistry results further showed that VEGF expression in the HIF-1α-VEGF siRNA group was weakly positive, while that in the HIF-1α siRNA group and VEGF siRNA group was positive. In addition, subsequently followed by the HIF-1α-VEGF siRNA group, the expression of VEGF and HIF-1α were similar in the RT-qPCR and Western blotting assays, and were both the lowest in the normal control group. VEGF is a crucial contributor to stimulating the growth of new vessel, and patients who are suffered from neovascular age-related macular degeneration (NVAMD), a branch of vascular diseases, have received substantial benefits of the research on special inhibitors of VEGF [27]. VEGF is mainly controlled by HIF-1α, a transcription factor that regulates hypoxia-inducible gene, and the reduced HIF-1α expression leads to the decreased VEGF expression [28]. Under hypoxic condition, the expression of VEGF is up-regulated by HIF-1α, which causes the increase in vascular permeability and retinal neovascularization, while the retinal neovascularization decreases due to the inhibition of HIF-1α [29]. These findings suggest that silencing of HIF-1α and VEGF occupy an important position in retinal neovascularization.

In conclusion, our results demonstrate that VEGF and HIF-1α gene silencing acts synergistically to inhibit alkali burn-induced CNV in rabbits and VEGF and HIF-1α gene silencing is expected to be a new treatment for CNV. However, the present study has several limitations. We do not make a further study on the mechanism of VEGF and HIF-1α gene silencing in rabbit corneal alkali burn, and therefore deeper study and discussion on the effects of VEGF and HIF-1α gene silencing based on downstream signaling pathway are needed in the future. CNV is a complicated process. At present, researches on CNV have obtained some encouraging achievements, but in order to fully understand the mechanisms of CNV, medical workers should continue to work hard.

## Abbreviations

CNV: corneal neovascularization
HE: Hematoxylin–Eosin
HIF: hypoxia-inducible factor
NC: negative control
RT-qPCR: reverse transcription quantitative PCR
VEGF: vascular endothelial growth factor
